The article "Comparison of Anterior Segment Optical Tomography Parameters Measured Using a Semi-Automatic Software to Standard Clinical Instruments" was published in 2013. Journal: PLoS One.

# Comparison of Anterior Segment Optical Tomography Parameters Measured Using a Semi-Automatic Software to Standard Clinical Instruments

**DOI:** 10.1371/journal.pone.0065559

**Published:** 2013-06-04

**Authors:** Marcus Ang, Wesley Chong, Huiqi Huang, Wan Ting Tay, Tien Yin Wong, Ming-Guang He, Tin Aung, Jodhbir S. Mehta

**Affiliations:** 1 Singapore National Eye Centre, Singapore, Singapore; 2 Singapore Eye Research Institute, Singapore, Singapore; 3 Department of Ophthalmology, National University Health System, Singapore, Singapore; 4 Centre for Eye Research Australia, University of Melbourne, Melbourne, Australia; 5 State Key Laboratory of Ophthalmology, Zhongshan Ophthalmic Center, Guangdong, China; 6 Department of Clinical Sciences, Duke-NUS Graduate Medical School, Singapore, Singapore; Justus-Liebig-University Giessen, Germany

## Abstract

**Objective:**

To compare anterior segment parameters measured using a semi-automatic software (Zhongshan Angle Assessment Program, ZAP) applied to anterior segment optical coherence tomography (AS-OCT) images, with commonly used instruments.

**Methods:**

Cross-sectional study of a total of 1069 subjects (1069 eyes) from three population-based studies of adults aged 40–80 years. All subjects underwent AS-OCT imaging and ZAP software was applied to determine anterior chamber depth (ACD), central corneal thickness (CCT), anterior and keratometry (K) – readings. These were compared to auto-refraction, keratometry and ocular biometry measured using an IOLMaster, ultrasound pachymeter and auto-refractor respectively. Agreements between AS-OCT (ZAP) and clinical instrument modalities were described using Bland-Altman, 95% limits of agreement (LOA).

**Results:**

The mean age of our subjects was 56.9±9.5 years and 50.9% were male. The mean AS-OCT (ZAP) parameters of our study cohort were: ACD 3.29±0.35 mm, CCT 560.75±35.07 µm; K-reading 46.79±2.72 D. There was good agreement between the measurements from ZAP analysis and each instrument and no violations in the assumptions of the LOA; albeit with a systematic bias for each comparison: AS-OCT consistently measured a deeper ACD compared to IOLMaster (95% LOA −0.24, 0.55); and a thicker CCT for the AS-OCT compared to ultrasound pachymetry (16.8±0.53 µm 95% LOA −17.3, 50.8). AS-OCT had good agreement with auto-refractor with at least 95% of the measurements within the prediction interval (P value <0.001).

**Conclusion:**

This study demonstrates that there is good agreement between the measurements from the AS-OCT (ZAP) and conventional tools. However, small systematic biases remain that suggest that these measurement tools may not be interchanged.

## Introduction

The anterior segment optical coherence tomography (AS-OCT) is increasingly being used to assess a number of common parameters of the anterior segment in various clinical settings. Anterior segment assessment is important for planning of surgical procedures. [1] Central corneal thickness (CCT) measurements are required for pre-operative evaluation for corneal refractive procedures. [2] Anterior chamber depth (ACD) calculations not only play a role in diagnosing mechanisms of glaucoma, but also in planning for surgical interventions such as phakic intraocular lens (IOL) implantations. [3] Moreover, ACD and corneal curvature with keratometry (K) - readings are important for IOL calculations. [4] Assessment of corneal curvature is also important in planning laser refractive surgery, orthokeratology therapy and fitting of contact lenses.

One of the limitations of AS-OCT is that there is no easy way to analyze the images rapidly and accurately. To address this gap, the Zhongshan Angle Assessment Program (ZAP, Guangzhou, China), a research, non-commercial software when applied to AS-OCT images, has been shown to reliably assess ACD and other anterior segment parameters. [5], [6], [7], [8], [9] Using gray-scale images, ZAP analyzes images by progressively tailoring contrast threshold and noise filters until a good pixel intensity distribution is achieved. With scleral spurs as points of reference, ZAP algorithms identify and define anatomical structures, deriving anterior segment measurements with high inter- and intra-observer agreement. [6], [7] Following the introduction of ZAP, AS-OCT images can be rapidly analyzed to provide an objective set of parameters for diagnosing and monitoring progress of various ocular diseases. [10], [11] However, whether the parameters assessed from ZAP are comparable with the same parameters measured from common clinical instruments is unclear.

The aim of this study was to compare the anterior segment parameters derived from rapid assessment of AS-OCT images using the ZAP software, with conventional methods of assessment such as ultrasound pachymetry or biometry. Our multi-racial population representing three major racial groups in Asia provides a unique opportunity to study these anterior segment parameters. [12].

## Methods

### Study Population

Our study subjects were recruited from the Singapore Epidemiology of Eye Disease Study, which comprises three population-based studies: the Singapore Malay Eye Study (SiMES, 2004–2006), the Singapore Indian Eye Study (SINDI, 2007–2009), and the Singapore Chinese Eye Study (SCES, 2009–2011). Details of the study methodologies are published elsewhere. [12], [13] All of these studies were conducted at the Singapore Eye Research Institute with approval from the Singhealth Institutional Review Board. They were conducted in accordance with the Declaration of Helsinki, with written informed consent obtained from all subjects before participation.

### Study Examinations

Ethnic Malays, Indians, and Chinese aged 40–80 years were randomly sampled to be included in each of these studies. For this particular study, we recruited subjects by systematically sampling (every fifth subject) who met the study eligibility criteria as described previously. [12] We excluded subjects with previous intraocular surgery or laser treatment, penetrating eye injury, or corneal disorders preventing anterior chamber assessment. A detailed interviewer-administered questionnaire was used to collect relevant socio-demographic data and medical history from all participants. In each study subject, auto-refraction, keratometry and ocular biometry were measured using an auto-refractor (Canon RK-5 Auto Ref-Keratometer, Canon Inc. Ltd., Japan) and the IOLMaster (Carl Zeiss; Meditec AG Jena, Germany) respectively – since the study is comparing anterior segment parameters, we will not report the other data derived from the IOLMaster. Central corneal thickness was measured using an ultrasound pachymeter (Advent, Mentor O&O, USA).

We prospectively performed consecutive, anterior segment scans of the right eye from each participant using the AS-OCT (Visante, Carl Zeiss Meditec, Dublin, CA) under standardized conditions of light (20 lux) by an operator who was masked to the results of the clinical ophthalmic examinations. [14] Scans were centered on the pupil and taken along the horizontal axis (nasal-temporal angles at 0–180 degrees) using the standard anterior segment single-scan protocol to maximize visibility of anatomic location and repeatability. [15] The ZAP software (research software, available upon request from the corresponding author, [none of the authors have any commercial interest]) was then used to assess all AS-OCT images using an algorithm previously described, [8] where the only observer input was to determine the location of the 2 scleral spurs in each image (WC). The scleral spur was defined as the anatomic junction between the inner wall of the trabecular meshwork and the sclera. [16] Briefly, the ZAP software automatically extracted the 300×600 8-bit grayscale (intensities from 0 to 255) image and produced a binary copy where pixels were either 1’s (tissue) or 0’s (open space) when compared to a calculated threshold value. Algorithms then used basic edge arguments (5 consecutive 0’s above, and 5 consecutive 1’s below indicated an anterior surface point) to describe the borders such as the corneal epithelium, endothelium and the anterior surface of the iris. These data were then fitted with polynomic curves and a line-smoothing algorithm to repair step-like portions of the border. The resultant data was then analyzed to derive the anterior segment and corneal parameters: ACD, CCT and keratometry (K) - readings. [6], [8] To compare ACD measurements from the IOLMaster to the AS-OCT, we added the ‘internal’ ACD (the aqueous depth) (posterior surface of cornea) to the CCT derived from the ZAP software. [17].

### Statistical Methods

All analyses were performed using SPSS version 20 (IBM Corp, Armank, NY). Mean with standard deviation (SD) were calculated for continuous anterior segment variables. Mean differences in measurements between groups were assessed using independent and paired samples t-tests, where appropriate. Biases (%) were calculated by dividing mean differences over means of the anterior segment parameters. Pearson correlation coefficients (*r*) were calculated to illustrate the strength of the linear relationship between various anterior segment parameters. Agreement between parameters from the ZAP AS-OCT images and the reference instruments was assessed using the method described by Bland and Altman, with 95% limits of agreement (LOA = mean difference ±1.96 SD) and its 95% confidence intervals calculated and assumptions checked. [18] All reported *p*-values were compared at a significance level of 5%.

## Results

A total of 1118 eyes (of 1118 subjects) were analyzed in our study, of which we obtained reliable anterior segment measurements from 1069 eyes (96%) (49 images did not have identifiable scleral spurs). The mean age of our subjects was 56.9±9.5 years and 50.9% were males. The demographics of our study subjects and their anterior segment parameters using each instrument are detailed in Table 1. The mean AS-OCT (ZAP) parameters of our study cohort were: ACD 3.29±0.35 mm, CCT 560.75±35.07 µm; K-reading 46.79±2.72 D.

**Table 1:** Characteristics of anterior segment parameters in study population.

Characteristics	Sub-category	*n*	ACD (mm)					CCT (µm)					K-reading (D)			
			AS-OCT (ZAP)			IOLMaster		AS-OCT (ZAP)			Ultrasound Pachymetry		AS-OCT (ZAP)		Auto Refractor	
			Mean	(SD)		Mean	(SD)	Mean	(SD)		Mean	(SD)	Mean	(SD)	Mean	(SD)
All persons		1069	3.29	(0.35)		3.13	(0.38)	560.75	(35.07)		544.00	(35.03)	46.79	(2.72)	43.98	(1.53)
Age	40–49	301	3.42	(0.33)		3.27	(0.37)	566.58	(37.31)		552.81	(37.48)	46.45	(2.26)	43.92	(1.49)
	50–59	363	3.31	(0.34)		3.17	(0.35)	561.79	(34.39)		544.94	(34.20)	46.50	(2.36)	43.91	(1.50)
	60–69	281	3.18	(0.36)		3.02	(0.37)	558.30	(33.36)		538.81	(32.58)	47.21	(3.05)	44.04	(1.56)
	≥70	124	3.14	(0.31)		2.93	(0.36)	549.10	(32.15)		531.60	(31.02)	47.54	(3.57)	44.20	(1.62)
	*P*-value for trend*		<0.001			<0.001		<0.001			<0.001		<0.001		0.255	
Gender	Male	544	3.35	(0.35)		3.19	(0.38)	559.22	(34.70)		542.78	(35.43)	46.48	(2.55)	43.69	(1.50)
	Female	525	3.22	(0.34)		3.07	(0.37)	562.33	(35.42)		545.27	(34.60)	47.12	(2.86)	44.28	(1.50)
	*P*-value*		<0.001			<0.001		0.147			0.245		<0.001		<0.001	
Race	Chinese	320	3.27	(0.33)		3.22	(0.34)	567.85	(33.43)		552.82	(35.14)	47.32	(2.14)	43.80	(1.54)
	Indian	496	3.28	(0.37)		3.07	(0.40)	561.81	(34.00)		538.83	(32.96)	47.31	(2.86)	44.11	(1.54)
	Malay	253	3.32	(0.34)		3.13	(0.37)	549.69	(36.58)		542.98	(36.77)	45.11	(2.42)	43.95	(1.47)
	*P*-value*		0.291			<0.001		<0.001			<0.001		<0.001		0.017	

* based on analysis of variance or independent-samples t-test where appropriate.

ACD: anterior chamber depth; CCT: central corneal thickness; K: keratometry; D: diopters; AS-OCT: anterior segment optical coherence tomography; ZAP: Zhongshan Angle Assessment Program; SD: standard deviation; n: number of subjects.

We summarized the anterior segment parameters comparing AS-OCT (ZAP) and the respective reference instruments in Table 2. We did not detect any violations in the assumptions of the limits of agreement – while the deviation of the mean difference from the zero-line in the Bland-Altman plots describes the presence of constant bias in all three comparisons. We found good agreement between the AS-OCT (ZAP) with the IOLMaster (at least 95% of all measurements were within the LOA), where a constant bias (mean difference 0.16 mm) was found as the AS-OCT consistently measured a deeper anterior chamber depth compared to the IOLMaster (95% LOA −0.24, 0.55) – Figure 1. This was similar to CCT measurements, where we found a good agreement between the AS-OCT and ultrasound pachymetry with 95% of measurements within the LOA (95% LOA −17.3, 50.8). There was an observed constant bias of 16.8±0.53 µm (3.03%) for the AS-OCT (ZAP) measuring a thicker CCT compared to ultrasound pachymetry– Figure 2.

**Figure 1:** Bland-Altman plot of anterior chamber depth (ACD) measurements, with zero-line (blue line), mean difference (red line) and 95% limits of agreement (green dotted lines), comparing AS-OCT (ZAP) and IOLMaster. X-axis units = mm/Y-axis units = mm.

**Figure 2:** Bland-Altman plot of central corneal thickness (CCT) measurements, with zero-line (blue line), mean difference (red line) and 95% limits of agreement (green dotted lines), comparing AS-OCT (ZAP) and Ultrasound Pachymetry. X-axis units = µm/Y-axis units = µm.

**Table 2:** Comparison of anterior segment parameters measured by anterior segment optical coherence tomography and various modalities.

Anterior segment parameters	Mean	Difference		Bias	*P*-value*	95% LOA		95% CI of LOA			
		Mean	(SD)					Lower LOA		Upper LOA	
ACD†(mm)	3.21	0.16	(0.20)	4.88%	<0.001	(−0.24,	0.55)	(−0.26,	−0.22)	(0.53,	0.57)
CCT (µm)	552.37	16.75	(17.35)	3.03%	<0.001	(−17.26,	50.76)	(−19.06,	−15.46)	(48.96,	52.56)
K-reading (D)	45.39	2.81	(2.36)	6.19%	<0.001	(−1.81,	7.43)	(−2.06,	−1.57)	(7.19,	7.68)

* based on paired-samples t-test.

† ACD measurements by ZAP have CCT measurements by ZAP added to allow comparison with ACD measurements by IOLMaster.

ACD: anterior chamber depth; CCT: central corneal thickness; K: keratometry; D: diopters; SD: standard deviation; LOA: limits of agreement; CI: confidence interval; ZAP: Zhongshan Angle Assessment Program.

In terms of K-readings, we found that there was good agreement as at least 95% of the data points were in prediction interval, with a proportional bias observed between the AS-OCT (ZAP) and the auto-refractor. The AS-OCT (ZAP) overestimated the K-readings compared to the auto-refractor by a mean of 2.81±2.36. The difference between the K-readings of the two methods was regressed on the average of K-readings of the two methods with its 95% prediction interval drawn – Figure 3. Table 3 describes the correlations for ACD, CCT and K-readings between AS-OCT (ZAP) and the reference instruments. While ACD and CCT had Pearson correlation coefficients of more than 0.85 (*p*-value <0.001), K-readings had a relatively lower Pearson correlation coefficient.

**Figure 3:** Bland-Altman plot of keratometric (K)-readings with the difference between the K-readings of the two methods regressed on the average of K-readings with its 95% prediction interval. X-axis units = D/Y-axis units = D.

**Table 3:** Correlations of anterior segment parameters measured by anterior segment optical coherence tomography and various modalities.

Anterior segment parameters	Measurement modality	Mean	(SD)	Pearson Correlation	*P*-value
ACD*(mm)	AS-OCT (ZAP)	3.29	(0.35)	0.85	<0.001
	IOL Master	3.13	(0.38)		
CCT (µm)	AS-OCT (ZAP)	560.75	(35.07)	0.88	<0.001
	Ultrasound Pachymetry	544	(35.03)		
K-reading (D)	AS-OCT (ZAP)	46.79	(2.72)	0.50	<0.001
	Auto Refractor	43.98	(1.53)		

* ACD measurements by ZAP have CCT measurements by ZAP added to allow comparison with ACD measurements by IOLMaster.

ACD: anterior chamber depth; AS-OCT: anterior segment optical coherence tomography; ZAP: Zhongshan Angle Assessment Program; CCT: central corneal thickness; K: keratometry; D: diopters; SD: standard deviation.

## Discussion

Although there were biases in the measurements, our study has demonstrated that the ZAP analyses of AS-OCT images produce measurements that are generally of good agreement with the reference instruments since at least 95% of the data points and differences were within the 95% prediction intervals and 95% LOA respectively. AS-OCT (ZAP) consistently measured a deeper ACD compared to IOLMaster (0.16±0.20 mm) and a thicker CCT compared to ultrasound pachymetry (16.8±0.53 µm). We also found that the AS-OCT (ZAP) had good agreement with auto-refractor measurements for K-readings, with at least 95% of the measurements within the prediction interval (P value <0.001). Using this population-based study we are able to describe the relationship between the results using the ZAP software on the AS-OCT scans, and each instrument.

The biases that we observed are likely due to either a fundamental difference in the principles of measurement between tools, or differences that have arisen from the actual analysis from the ZAP software. However, the aim of this study was not to determine why these observed differences exist, or if any one tool is superior – but instead, to demonstrate the usefulness of a rapid diagnostic software which may be used for AS-OCT image analysis and how the parameters compare to conventional tools used in our daily clinical practice. The ZAP software works by extracting the gray-scale images from the AS-OCT images and uses image processing and algorithms to define the anatomical landmarks, which has been described in detail before. [6] It then uses the observer input of scleral spurs as points of reference, with other anatomical points such as the borders of the cornea endothelium and anterior surface of the iris, to objectively derive the other corneal parameters. [6] This allows for potential reduction in inaccuracies that can arise from subjective placement of the measurement tools on the AS-OCT image.

Accurate ACD measurements are important for accurate biometric calculations, surgical planning and predicting risk of diseases such as angle closure. Previous studies have shown that anterior segment measurements using the AS-OCT are highly reproducible and show good repeatability, compared to the IOLMaster. [19], [20], [21] However, measurements of the ACD from AS-OCT images still remains relatively subjective as it is evaluated using a caliper or white-to-white measurements. [21] The ZAP software now allows for a more objective measurement of ACD, albeit with a constant bias of a deeper anterior chamber (mean 0.16 mm) compared to IOLMaster. [22] It has been suggested that the AS-OCT produces a more accurate measurement of ACD, as the AS-OCT does not affect the state of accommodation, and has less effect on pupil size. [19] Our study also confirms that ACD decreases with age, is shallower in females compared to males and is smallest in Chinese compared to Malays and Indians. [23] Although both AS-OCT images and IOLMaster measurements are obtained using similar principles of Michelson interferometry, ACD differences and thus biases, may arise due to different wavelengths that AS-OCT (1310 nm) and IOLMaster (780 nm) use.

Together with ACD, CCT is a clinically important parameter in the diagnosis of glaucoma, [24] as well as planning for refractive procedures such as LASIK. Previous studies have found a difficulty in determining the CCT from AS-OCT - either underestimating as the calipers are placed slightly below the true anterior corneal surface; or overestimating with calipers that are manually placed on the anterior corneal surface. [25] Using the ZAP software, we are able to more objectively measure CCT from AS-OCT images rather than rely on manual placement of calipers, which may lead to an underestimation of CCT as compared to ultrasound pachymetry as reported in a previous study. [26] However, ultrasound pachmetry is a contact method, which will inadvertently cause axial compression of the cornea, and could also result in underestimation of the actual true central corneal thickness. This may explain the results of our study where we observed that the AS-OCT (ZAP) consistently measured a thicker CCT (mean 16.8 µm) as compared to ultrasound pachymetry.

Keratometry, another important parameter used in IOL calculation, could also be directly calculated from AS-OCT using the ZAP software. Our population-based study demonstrated that despite the generally good agreement between AS-OCT measurements and the auto-refractor, there exists a proportional bias. This means that the AS-OCT may measure a lower K-reading compared to the auto-refractor for lower readings (lowest quartile, mean difference: 1.42±2.26); and a higher reading for measurements in the upper range (highest quartile, mean difference: 4.25±2.92). This may be due to differences in the way each tool makes the measurements: unlike the auto-refractor which assumes the cornea to be a convex mirror and uses reflected corneal mires to compute the radius of corneal curvature, the AS-OCT (ZAP) objectively measures the anterior and posterior corneal curvatures to derive the keratometry readings. [17] Moreover, keratometry readings from ZAP are derived based on corneal curvature derived from algorithms of AS-OCT images in a single horizontal plane. This could explain the difference in readings from the auto-keratometer, where K-readings are geometrically derived from manipulating rays in two planes.

The inability to detect the scleral spur, in suboptimal images and where the sclera formed a smooth continuous line, is another recognized limitation in all studies involving ZAP. However, we were able to reliably measure 96% of all our AS-OCT scan images. The advantage of the ZAP software is that once these scleral spurs are identified, the rest of the measurements are produced automatically. Only horizontal nasal–temporal AS-OCT scans were used, as these have been shown to be the most consistent with respect to obtaining high-quality images for the ZAP software to analyze. However, this ensured that there was a very high rate of scleral spur visibility and thus more valid scans, compared to if we had chosen vertical scans. [16].

In conclusion, we found a good agreement between the anterior segment parameters from AS-OCT ZAP analyses with conventional instruments. However, small systematic biases remain which suggest that these measurement tools may not be interchanged. Nevertheless, with further modifications, our study suggests that semi-automated software such as ZAP, applied to AS-OCT imaging, may improve the usability of a single imaging device to assess a set of anterior segment parameters in an objective way.
